# Green Human Resource Management, Employee Work Values, and Enterprise Environmental Performance

**DOI:** 10.1155/2022/8129359

**Published:** 2022-06-27

**Authors:** Junyan Liu, Yongli Wu

**Affiliations:** Krirk University, No. 3 Soi Ramintra 1, Ramintra Road, Anusaowaree, Bangkhen, Bangkok 10220, Thailand

## Abstract

China's economy is developing rapidly, and enterprises are paying more and more attention to environmental protection in the process of economic development. However, relatively speaking, the environmental awareness of enterprises and employees needs to be further improved. This paper investigates the impact of green human resource management on environmental performance by questionnaire survey. A total of 372 questionnaires were distributed to front-line employees and human resource supervisors, 357 of which were valid. Using descriptive statistics, correlation analysis, regression analysis, and mediating effect test, this paper studies the relationship between green human resource management and environmental performance, and tests the mediating role of employees' work values between green human resource management and enterprise environmental performance. The conclusion of the empirical study has some inspiration for the green human resource management of enterprises, provides some references for the development of relevant theories, and provides practical significance for the green development of enterprises.

## 1. Introduction

Enterprise green human resource management has a positive impact on employees' values and norms of behavior in daily work. The realization of the strategic goal of sustainable development is closely related to the resources the enterprise has, and this “resource” is every employee in the enterprise. Wang [1] proposed that human resource management departments can make full use of the balance of human resource protection and vigorously promote green management among employees. While mobilizing employees' subjective initiative, let each employee devote himself to daily work with a positive attitude. Pan 'e and Guo [2] proposed energy-saving and emission reduction, reducing pollution and waste, and the new idea of harmonious coexistence of the natural environment is implemented in every corner of the enterprise. Richa [3] conducted a comprehensive study on green human resources management and enterprise and analysed the influence of the environmental performance, and considered employee work value as an intermediary variable to study the effect of green human resource management on the environmental performance for the analysis of the specific human resources in enterprises through research, and summed up the green environmental protection performance and the role and significance. In the following sections, I will carry out a literature review and provide hypothesis, research methods, data analysis, results, and discussion.

## 2. Research Hypotheses and Research Models

### 2.1. Related Research and Hypothesis

Ren et al. [4] believe that employee system management in enterprises is an important cornerstone for the popularization of environmental protection behavior in enterprises, and the attention and support from leaders greatly affect employees' attitudes towards environmental protection activities. Yang [5] showed that corporate leaders' attention to environmental protection would affect employees' awareness and behavior of environmental protection at work. Therefore, this study divides employee system management into the formalization of enterprise environmental protection regulations, integration degree of employee regulations, and attention and support from leaders, so as to interpret the impact of green human resource management on enterprise environmental protection performance.

Tang et al. [6] believe that by implementing green human resource management in enterprises, employees can reduce waste in the production process, and rationally utilize resources. Zhou and Zhang [7] reduce resource consumption, reduce the damage to the natural environment through the processing of sewage and pollutants, and ultimately improve the environmental performance of enterprises. Qian and Zhang [8] proposed that the environmental consciousness of employees is divided into employee pollution control consciousness and employee pollution prevention consciousness.

Wang et al. [9] believe that employees working in different organizational cultures will have different work values and thus affect their work behaviors. Ogbeibu et al. [10] proposed that employees are sensitive to green human resource management to different degrees under the guidance of different values. Dumont et al. [11] measured the impact of green human resource management on work and employees' lives from a six-item scale of four dimensions. Saeed et al. [12] and Yong et al. [13] divide green human resource management into five dimensions. This paper uses 10 items of five dimensions for measurement. In this paper, employees' work values as intermediary variables, green enterprise human resource management, and employee two-way interactive process were studied. Green enterprise human resource management for employees to perceive the extent of the environmental protection, motivation of employees to choose to participate in the organization to work for environmental protection, and promotion of the smooth implementation of enterprise environmental management measures were studied. Therefore, we propose the following hypothesis:

H1: Green human resource management has a positive impact on enterprise environmental performance.
H2: Employee system management has a positive impact on enterprise environmental performance.
    H2-1: Formalization of enterprise environmental regulations has a positive impact on enterprise environmental performance.
    H2-2: The integration degree of employee regulations has a positive impact on enterprise environmental performance.
    H2-3: Attention and support from leaders have a positive impact on enterprise environmental performance.
H3: Employees' environmental awareness has a positive impact on enterprise environmental performance.
    H3-1: Employees' awareness of pollution control has a positive impact on enterprise environmental performance.
    H3-2: Employees' awareness of pollution prevention has a positive impact on enterprise environmental performance.
H4: Employees' work values have a mediating effect on green human resource management and enterprise environmental performance.

### 2.2. Technology Roadmap

This paper mainly studies the impact of green human resource management on environmental performance. Green human resource management is divided into two dimensions, namely, employee system management and employee environmental awareness, and the impact of green human resource management on environmental performance is studied by taking the employee work value as an intermediary variable. The technical route is shown in Figure 1.

## 3. Methods

### 3.1. Research Tools

Based on the reference of the literature, this study compiled questionnaires and collected data by using a questionnaire survey. Likert 5-scale was used for measurement, with scores ranging from “1” to “5” representing from “completely inconsistent” to “completely consistent.” The responses were very consistent = 5; in line with the = 4; generally = 3, not = 2; it is very inconsistent with = 1.

### 3.2. Samples and Data Collection

The selected samples come from 53 enterprises in The Beijing-Tianjin-Hebei region, involving the domestic service industry, manufacturing industry, construction industry, and logistics. Front-line employees and human resource supervisors of enterprises are taken as research objects in the survey. 372 formal questionnaires were sent out, and 365 were recovered, with 357 valid questionnaires and an effective recovery rate of 95%. Among them, 45.65% are male, 54.34% are female, 73.1% are ordinary employees, and 57.98% are with a bachelor's degree. The manufacturing industry accounted for 32.07%, service industry 20.75%, construction industry 26.41%, and logistics industry 20.75%. The types of enterprises are mainly the manufacturing industry, service industry, construction industry, and logistics industry, accounting for 32.07%, 20.75%, 26.41%, and 20.75%, respectively.

## 4. Data Analysis

In this paper, SPSS23.0 was used to test the reliability and validity of the questionnaire data. The reliability of the total table of green human resource management and the second-level dimensions were all above 0.8, the KMO value was greater than 0.7, and both were significant at the level of 0.001. The reliability and structural validity were good and could be used in the study.

### 4.1. Descriptive Statistical Analysis of Each Variable

Conduct descriptive statistics on the overall score of green human resource management and five dimensions (see details in Table 1).

As shown in Table 1, the overall score of green human resource management is 3.82, 3.65, 3.68, 3.13, and 3.54, respectively, for the formalization of enterprise environmental protection regulations, the integration degree of employee regulations, the attention and support of leaders, the awareness of employee pollution control, and the awareness of employee pollution prevention. The overall score of green human resource management is 3.56. Overall, the scores of employees' pollution control consciousness and pollution prevention consciousness are lower than the overall score of green human resource management, and the scores of formalization of enterprise environmental protection regulations, integration of employees' regulations, and attention and support from leaders are higher than the overall score of green human resource management.

### 4.2. Correlation Analysis

Test the correlation between the five dimensions of green human resource management and environmental performance (see details in Table 2).

As shown in Table 2, in the correlation test, the formalization of enterprise environmental protection regulations, the integration degree of employee regulations, the attention and support of leaders, the awareness of employee pollution control, and the awareness of employee pollution prevention and environmental protection performance all have a significant positive correlation at the level of 0.01. The correlation coefficients were 0.386, 0.427, 0.512, 0.501, and 0.413, respectively.

### 4.3. Research on the Impact of Green Human Resource Management on Environmental Performance

Five dimensions of green human resource management were taken as predictive variables and environmental performance as dependent variables to conduct the regression model test (see details in Table 3).

As shown in Table 3, linear regression was used to test the regression model, and the formula was as follows: environmental performance = 0.214^*∗*^ formalization of enterprise environmental protection regulations +0.083^*∗*^ integration of employee regulations +0.207^*∗*^ attention and support from leaders +0.231^*∗*^ awareness of employee pollution control +0.171^*∗*^ awareness of employee pollution prevention +0.561 in the regression model test of formalization of enterprise environmental protection regulations, integration degree of employee regulations, attention and support from leaders, awareness of employee pollution control and awareness of employee pollution prevention on environmental protection performance, the regression model (*F* = 68.054, ^*∗*^) is significant at 0.001 level, that is, the regression model is effective at 0.001 significance level, *R*^2^ = 0.492, that is, the independent variable can explain 49.2% of the variation of the dependent variable.

In the significance test of regression coefficient, the enterprise environmental protection regulations were formalized (*b* = 0.214, *t* = 5.158, *P* < 0.001), employee regulation integration (*b* = 0.083, *t* = 2.300, *P* < 0.05), leadership attention and support (*b* = 0.207, *t* = 6.455, *P* < 0.001), employee awareness of pollution control (*b* = 0.231, *t* = 6.191, *P* < 0.001), and employee awareness of pollution prevention (*b* = 0.171, *t* = 4.938, *P* < 0.001) have positive prediction effect on environmental performance, that is, the higher the score of formalization of enterprise environmental regulation, the integration degree of employee regulation, the attention and support of leaders, the higher the score of employee pollution control consciousness and employee pollution prevention consciousness, and the higher the score of environmental performance. The lower the score of formalization of enterprise environmental protection regulations, integration of employee regulations, attention and support from leaders, awareness of pollution control and awareness of pollution prevention, and the lower the score of environmental protection performance.

In conclusion, the formalization of enterprise environmental regulations, the integration degree of employees' regulations, the attention and support of leaders, the awareness of pollution control of employees, and the awareness of pollution prevention of employees have a significant positive impact on environmental performance, among which the attention and support of leaders have the greatest impact. The second is the employee pollution control consciousness, enterprise environmental protection regulation formalization, employee pollution prevention consciousness, employee pollution prevention consciousness, and employee regulation integration degree.

### 4.4. The Mediating Effect of Employee Work Values

Taking green human resource management as the independent variable, environmental performance as the dependent variable, and employees' work values as the mediating variable, the mediating effect test was conducted (see details in Table 4).

As can be seen from Table 4, in the test of mediating effect of employee work values on green human resource management and environmental performance, *C* = 0.885, significant at 0.001 level; *A* = 0.289, significant at 0.001 level; *B* = 0.725, significant at 0.001 level; Kede employees' work values play an intermediary role between green human resource management and environmental performance. *C*' = 0.675, significant at 0.001 level. To sum up, the employee's work values have a partial mediating effect between green human resource management and environmental performance, the mediating effect = (0.289^*∗*^0.728)/0.885 = 23.68%.

## 5. Research Results and Discussion

### 5.1. Study Results

This paper verifies the relationship between green human resource management and enterprise environmental performance through regression analysis, and obtains the following results: green human resource management has a positive effect on enterprise environmental performance; employee's work values play a partially mediating role in green human resource management and enterprise environmental performance. So far, all the hypotheses in this study have been tested, and the results of hypothesis testing are summarized in Table 5.

### 5.2. Discussion

Through empirical tests, enterprises improve the quality of employees, strengthen pollution prevention and control, pay attention to management methods, and create a good environment for the implementation of green human resource management by integrating management capabilities and support, thus having a positive role in promoting environmental performance. Hypothesis H1 is established. The green employee system management enhances employees' awareness of environmental protection, urges employees to attach importance to environmental protection behaviors, and has a positive impact on environmental performance. Hypothesis H2 is established. Formalized incorporation of enterprise environmental protection regulations into the employee system management will enhance employees' environmental protection behavior and thus have a positive impact on environmental protection performance, assuming H2-1 is true. Alkhateeb et al. [14] proposed that when leaders attach importance to and support the employee system management integrated with employee regulations as the purpose of the enterprise, employees' environmental awareness will gradually improve on the original basis. Therefore, H2-2 and H2-3 are assumed to be established. Richa [3] proposed that when the enterprise promotes employee system management and when the leaders can attach importance to and support all departments to take environmental protection factors into consideration in the goal or decision-making, it will promote the improvement of the environmental awareness of employees.

In the regression analysis, the higher the score of employees' pollution control awareness and pollution prevention awareness, the higher the score of environmental performance. Therefore, Saeed et al. [12] employees' environmental awareness has a positive impact on environmental performance. Hypothesis H3 is established. Green human resource management helps enterprises to establish employees' awareness of environmental protection and enhance their awareness of pollution control and prevention at work, thus having a positive impact on enterprise environmental performance. Hypothesis H3-1 and H3-2 are established.

In the test of mediating effect, employees' work values play a partial mediating role in green human resource management and enterprise environmental performance, and hypothesis H4 is established. Part of the impact of green human resource management on the company's environmental performance is conducted through employees' work values. Green human resource management can promote the improvement of employees' work values, and the improvement of employees' work values is conducive to the improvement of enterprise environmental performance, and the employee's work values play a partial intermediary role in the relationship between green human resource management and enterprise environmental performance.

### 5.3. Deficiencies and Prospects of Research

Despite the benefits yielded by this study, some limitations were encountered. First, the selection of samples in this paper may not be adequately comprehensive. The limited sample may lack a wholesome representation of companies. Second, this paper does not classify industries in the research process; therefore, different industries can be selected for comparative research in the future. Thirdly, this paper studies the mediating role of employees' work values in the relationship between green human resource management and corporate environmental performance. Additional mediating variables can be selected for more comprehensive studies.

## Figures and Tables

**Figure 1:** Technology roadmap.

**Table 1:** Descriptive statistics of each variable.

Variable	The minimum value	The maximum	The mean	The standard deviation
Formalization of environmental protection regulations for enterprises	1.88	5.00	3.82	0.63
Employees prescribe integration	1.20	5.00	3.65	0.78
Leadership attention and support	1.50	5.00	3.68	0.83
Employee awareness of pollution control	1.63	5.00	3.13	0.70
Awareness of employee pollution prevention	1.50	4.50	3.54	0.72
Green HUMAN resource management overall	2.04	4.45	3.56	0.47

Source: SPSS23.0 descriptive statistics.

**Table 2:** Correlation.

	Formalization of environmental protection regulations for enterprises	Employees prescribe integration	Leadership attention and support	Employee awareness of pollution control	Awareness of employee pollution prevention
Formalization of environmental protection regulations for enterprises	1				
Employees prescribe integration	0.468^*∗∗*^	1			
Leadership attention and support	0.166^*∗∗*^	0.382^*∗∗*^	1		
Employee awareness of pollution control	0.156^*∗∗*^	0.241^*∗∗*^	0.382^*∗∗*^	1	
Awareness of employee pollution prevention	0.125^*∗*^	0.220^*∗∗*^	0.252^*∗∗*^	0.331^*∗∗*^	1
Environmental performance	0.386^*∗∗*^	0.427^*∗∗*^	0.512^*∗∗*^	0.501^*∗∗*^	0.413^*∗∗*^

^*∗∗*^At 0.01 level (double-tailed), the correlation was significant. ^*∗*^At level 0.05 (two-tailed), the correlation was significant. Data source: collated according to the results of SPSS23.0 operation.

**Table 3:** Regression model test.

Model	Unnormalized coefficient		Normalization coefficient	*t*	Significance
	*B*	The standard error	Beta		
(Constant)	0.561	0.186		3.015	0.003
Formalization of environmental protection regulations for enterprises	0.214	0.042	0.222	5.158	0.000
Employees prescribe integration	0.083	0.036	0.106	2.300	0.022
Leadership attention and support	0.207	0.032	0.282	6.455	0.000
Employee awareness of pollution control	0.231	0.037	0.265	6.191	0.000
Awareness of employee pollution prevention	0.171	0.035	0.202	4.938	0.000
*R* ^2^	0.492				
*F*	68.054				0.000

Data source: collated according to the results of SPSS23.0 operation.

**Table 4:** Mediating effect test of employees' work values.

	Normalized regression equation	Regression coefficient test	
Step 1 (c)	*Y* = 0.885*X*	SE = 0.049	*t* = 18.079^*∗∗∗*^
Step 2 (a)	*M* = 0.289*X*	SE = 0.046	*t* = 6.275^*∗∗∗*^
Step 3 (b,c')	*Y* = 0.725*M*	SE = 0.041	*t* = 17.595^*∗∗∗*^
	+0.675*X*	SE = 0.038	*t* = 17.579^*∗∗∗*^

**Table 5:** Hypothesis testing results.

Assumption number	Assuming that the content	The inspection results
H1	Green human resource management has a positive impact on enterprise environmental performance	Support
H2	Employee system management has a positive impact on enterprise environmental performance	Support
H2-1	The formalization of enterprise environmental regulation has a positive influence on enterprise environmental performance	Support
H2-2	The degree of employee regulation integration has a positive impact on enterprise environmental performance	Support
H2-3	Leadership attention and support have a positive impact on enterprise environmental performance	Support
H3	Employee environmental awareness has a positive influence on enterprise environmental performance	Support
H3-1	Employees' awareness of pollution control has a positive influence on enterprise environmental performance	Support
H3-2	Employees' awareness of pollution prevention has a positive influence on enterprise environmental performance	Support
H4	Employees' work values have a mediating effect on green human resource management and enterprise environmental performance	Support

## Data Availability

All the data used in this study can be accessed by request.
